This article has been retracted.

# Postoperative Adjuvant Chemoradiotherapy on the Survival of Stage III Gastric Cancer

**DOI:** 10.1155/2022/8036763

**Published:** 2022-06-28

**Authors:** Chao Li, Shoupeng Shao, Yue Sun, Fujun Shen, Meijuan Wang, Hongsheng Wang, Chunbin Wang

**Affiliations:** Department of Oncology, Yancheng Third People's Hospital & The Sixth Affiliated Hospital of Nantong University, Yancheng, Jiangsu Province 224008, China

## Abstract

**Objective:**

Although adjuvant therapy has been shown to be beneficial in gastric cancer, the use of adjuvant chemoradiotherapy remains controversial. This paper investigated the effects of postoperative adjuvant chemoradiotherapy on the survival of patients with stage III gastric cancer.

**Methods:**

In total, the data of 72 stage III gastric cancer patients treated at our hospital from January 2014 to December 2019 were retrieved and assessed. They were categorized into a chemotherapy group (CT group) and a radiochemotherapy group (RCT group) according to their given treatment regimens. A 3-year follow-up was conducted to record their incidence of disease-free survival (DFS), overall survival (OS), and adverse events.

**Results:**

For the CT and RCT groups, DFS was 86.4% and 92.6% in the first year, decreasing to 55.1% and 73.7% in the second year, and 41.3% and 69.1% in the third year. There was no significant difference in DFS between the two groups during the three-year follow-up. Additionally, for the CT and RCT groups, their respective 1-year, 2-year, and 3-year OS were 95.6% and 96.3%, 75.1% and 87.9%, and 50.3% and 74.2%, indicating that the OS of patients in the RCT group was significantly higher than that in the CT group during 3 years of follow-up. Further, no significant difference in the incidence of adverse events was found between the two treatment groups.

**Conclusions:**

Collectively, adjuvant radiochemotherapy after radical gastrectomy for stage III gastric cancer was associated with better survival outcomes than chemotherapy, without increase in adverse events.

## 1. Introduction

As one of the most prevalent cancers, gastric cancer refers to a common malignant tumor in the digestive tract which originates from the epithelium and is one of the leading causes of cancer-related death worldwide [1, 2]. Due to the lack of early symptoms, most patients with gastric cancer, upon being diagnosed, are at the advanced stage (stage II, III, or IV) or locally advanced stage, accompanied by lymph node or distant organ metastasis and thus have poor prognoses [3, 4].

Currently, the 5-year survival rates of stage II, IIIA, IIIB, and IV gastric cancer patients are reported to be approximately 34%, 20%, 8%, and 7%, respectively. Radical resection remains the primary treatment for gastric cancer [5]. The postoperative 5-year survival rate is as high as 90% in patients with early gastric cancer, but in patients with advanced-stage disease, radical resection only is associated with a high risk of recurrence [6]. Further, it was reported that 40%-65% of radically resected patients could have local recurrences on the initial tumor bed, anastomotic region, or locoregional lymph nodes [7]. Metastasis is the predominant cause of poor treatment outcomes and mortality in gastric cancer, for which surgery and radiotherapy remain the only local treatments. Therefore, adjuvant therapy, including radiotherapy, intraperitoneal chemotherapy, immunochemotherapy, chemotherapy alone, and radiochemotherapy, are usually considered to improve the survival of these patients despite radical resection [8].

Adjuvant therapy in the treatment of gastric cancer has been shown to reduce the risk of mortality by 16% to 28%. In patients with IB or even higher, studies have shown that adjuvant therapy was undoubtedly necessary to decrease their risk of recurrence [9, 10]. In regard to adjuvant chemotherapy, its added value in postoperative treatment following gastrectomy was reported in several meta-analyses [11, 12]. Further, the value of adjuvant radiotherapy applied postoperatively has also been confirmed by relevant studies. The INT-0116 study reported the benefit of adjuvant concomitant chemoradiotherapy in improving the survival rate of gastric cancer patients [13]. However, not all patients underwent D2 curative radical gastrectomy.

Radiotherapy as a local treatment has been shown to be effective in terms of local control [14]. Previous clinical trials which compared adjuvant CT alone with RCT in gastric cancer and a meta-analysis consisting of 3 randomized clinical trials showed that although both treatments were well-tolerated and had an equally beneficial impact on the survival of the patients, there was no significant difference in distance relapse or overall survival [15]. Further, some oncologists believe that adjuvant radiotherapy could be associated with an increased risk of leakage, especially at the anastomotic site of the gastroesophageal junction [16]. Thus, the role of adjuvant chemoradiotherapy in the treatment of gastric cancer after surgery is still controversial [17].

This study is aimed at investigating the therapeutic effects and impact of adding postoperative radiotherapy on the survival of patients with stage III gastric cancer, compared to chemotherapy only, in an effort to lay a theoretical basis for the adjuvant clinical treatment of advanced gastric cancer.

## 2. Materials and Methods

### 2.1. Study Subjects

A total of 72 patients with stage III gastric cancer who received radical resection at our hospital from January 2014 to December 2019 were divided into a chemotherapy group (CT group, *n* = 45) and a radiochemotherapy group (RCT group, *n* = 27) based on the postoperative treatment they received. Inclusion criteria were (1) pathologically diagnosed as gastric/gastroesophageal junction adenocarcinoma; (2) postoperative stage III with an ECOG score of 0-2 points; (3) absence of liver, kidney, and bone marrow dysfunction; and (4) not received radiochemotherapy before and absence of other malignant tumors. Exclusion criteria were (1) presence of severe cardiovascular disease or respiratory disease; (2) diagnosed with uncontrolled diabetes, upper gastrointestinal obstruction, perforation or bleeding, or severe infection demanding treatment; and (3) had mental disorders or other solid tumors.

Informed consent was obtained from all patients, and the study was approved by the Ethics Committee of Yancheng Third People's Hospital (2020-13).

### 2.2. Treatment Regimens

After 4 weeks following surgery, all patients in the CT group were treated with adjuvant SOX (S-1 + oxaliplatin) or XELOX (capecitabine + oxaliplatin) regimen. The treatment was repeated every 3 weeks for 6 cycles.

In the RCT group, the lesions were routinely positioned using a BrightSpeed CT simulator. Radiotherapy was performed using a Varian linear accelerator (23-EX, UNIQUE), with a total radiation dose of 45-50.4 Gy (1.8-2 Gy per fraction, totally: 25-28 fractions). During radiotherapy or 2-3 weeks following radiotherapy, SOX or XELOX regimens were applied.

During the treatment, patients in both groups received adjuvant therapy, including nutrition, acid suppression, and gastric mucosal protective agent.

### 2.3. Outcome Measures

Blood routine tests, detection of liver and kidney function and gastrointestinal tumor markers, electrocardiogram, chest radiography, upper abdominal color ultrasound, and computed tomography were performed in each patient before treatment. All patients underwent a blood routine test once a week, and adverse reactions were evaluated during each treatment cycle. Toxicity above grade 4 would lead to the termination of concurrent radiochemotherapy. The grading of adverse reactions ranged from 1 to 5 according to CTCAE 5.0.

### 2.4. Follow-Up

After treatment, the patients were followed up for 3 years and information on survival status, overall survival (OS), and disease-free survival (DFS) rates were recorded.

### 2.5. Statistical Methods

All data were analyzed using the SPSS 25.0 software. Measurement data were expressed as mean ± standard deviation (mean ± SD), and a *t*-test was used for comparison between groups. Enumeration data were expressed as frequency (*n*) and percentage (%), and the cases were compared using the chi-square test. DFS and OS were calculated using the Kaplan-Meier method, and *p* < 0.05 was used as the reference for statistical significance.

## 3. Results

### 3.1. Baseline Characteristics of the Patients

In total, 72 patients, including 58 males and 14 females, aged 35-76 years old, were eligible for this study. Among them, 70 had lymph node invasion or metastasis. The CT group contained 45 patients (33 males and 22 females), with an average age of 58.57 ± 8.30 years. There were 27 patients in the RCT group, including 25 males and 2 females, with an average age of 60.33 ± 8.8 years old. No significant differences were observed in terms of age and clinical stage (Table 1) between the two groups, indicating relatively balanced cohorts.

### 3.2. Comparison of Incidence of Adverse Reactions between the Two Groups

Following statistical results of the incidence of adverse reactions after postoperative adjuvant treatment in the two groups, our results showed that most adverse events were of grades 1 and 2, and the most commonly observed adverse reactions were myelosuppression, gastrointestinal reactions (nausea, vomiting, etc.), neurotoxicity (hand-foot syndrome), and liver dysfunction. After further calculation, compared with the CT group, the RCT group had lower incidences of gastrointestinal reactions (92.6% vs. 60%), myelosuppression (85.1% vs. 73.3%), neurotoxicity (62.9% vs. 37.78%), and liver dysfunction (48.1% vs. 42.22%). There was no significant difference in the incidence of adverse reactions between the two groups (Table 2).

### 3.3. Comparison of Survival Rate between the Two Groups

After the 3-year follow-up, our results showed that the 1-year DFS was 86.4% and 92.6%, 2-year DFS was 55.1% and 73.7%, and 3-year DFS was 86.4% and 92.6% for the CT and RCT groups, respectively. The OS was 95.6% and 96.3% in the first year for the CT and RCT groups, which decreased to 75.1% and 87.9%, in the 2nd year, and was 50.3% and 74.2% in the third year. Taken together, the results showed that the DFS and OS of the RCT group were significantly higher than the CT group (Figure 1).

## 4. Discussion

With an alarming global prevalence and mortality rate, gastric cancer is one of the deadliest cancers [18]. In China, 70.8% of the cases are stage II-III gastric cancer, while stage I and IV gastric cancer accounts for 19.5% and 9.7% of all cases [19, 20]. Progressive gastric cancer refers to stage II-III gastric cancer, and advanced stages refer to cases with the invasion of cancer cells into the gastric wall and serosal layer, usually accompanied by lymph node, peritoneal, or hematogenous metastasis. Surgical resection of the primary tumor and regional lymph nodes constitutes the key treatment of gastric cancer. In Japan and Korea, D2 radical gastrectomy is the standard treatment for locally advanced gastric cancer, but due to the differences in surgical equipment in different regions, the surgical outcomes vary [21]. In addition, patients with advanced gastric cancer are prone to recurrence after receiving radical resection alone.

In this study, the baseline characteristics between the study patients were comparable in terms of gender, age, TNM stage, and ECOG score, suggesting homogeneity between the two treatment cohorts. We also found that the addition of radiotherapy to chemotherapy was beneficial in increasing the survival of the patients compared with chemotherapy only. These findings are concordant with previous studies. Kantzou et al. [16] reported that the combination of modern radiotherapy techniques with chemotherapy could improve treatment outcomes and be safe. Min et al. [22] peroformed a meta-analysis of randomized trials by comparing the efficacy of adjuvant CT with RCT, which comprised 1171 patients. They found that although there was no significant difference in OS between the 2 groups (odds ratio 1.27, 95% confidence interval 0.95-1.71), RCT was associated with higher DFS compared to CT alone (odds ratio 1.48, 95% confidence interval 1.08-2.03). Compared with our findings, our results showed that for the CT and RCT groups, the DFS was 86.4% and 92.6% in the first year, 55.1% and 73.7% in the second year, and 41.3% and 69.1% in the third year, indicating the RCT was significantly higher 1-year, 2-year, and 3-year DFS. However, compared to the study of Min et al. [22], our results showed that RCT was still associated with higher 1-year, 2-year, and 3-year OS than the CT group, especially from the second year after surgery, whereby for the CT and RCT groups, their respective 1-year, 2-year, and 3-year OS were 95.6% and 96.3%, 75.1% and 87.9%, and 50.3% and 74.2%.

Radiotherapy, as a local treatment, is an important supplement to surgery. Adjuvant radiochemotherapy is also recommended in CSCO guidelines [23, 24] as an option for stage III cancer. Adjuvant chemotherapy is currently the most commonly used therapy in the adjuvant treatment of locally advanced gastric cancer. The ACTS-GC and CLASSIC clinical trials showed that adjuvant chemotherapy (S-1/XELOX) after D2 gastrectomy was associated with a significantly reduced risk of death and prolonged survival length compared with surgery alone [25, 26]. The results of the INT 0116 study conducted in the United States showed that postoperative adjuvant radiochemotherapy could improve the survival rate of patients threatened by recurrence [27]. A 2014 study including 6 randomized controlled clinical trials involving 1171 gastric cancer patients with complete resection suggested that adjuvant radiochemotherapy performed better in terms of DFS than chemotherapy alone after surgery [22]. Consistently, our study showed that postoperative adjuvant chemotherapy significantly improved the DFS and OS of patients with gastric cancer.

In a recent ARTIST-II study, although adjuvant radiochemotherapy failed to improve the survival to a higher degree compared with adjuvant chemotherapy, it was associated with a decrease in local recurrence rate from 13% to 7% [28]. In terms of adverse reactions, the addition of adjuvant chemoradiotherapy did not effectively reduce the incidence in patients with stage III gastric cancer, which may be possibly due to the poor tolerance of patients to radical resection and adjuvant therapy. However, in this study, we observed that most of the adverse events were grade 1 and 2 adverse events, and there was no significant difference in the incidence of adverse events compared with the CT group.

## 5. Conclusion

This study found that postoperative adjuvant chemoradiotherapy was associated with improved 3-year OS and 3-year DFS, compared with adjuvant chemotherapy only, without any difference in adverse events in stage III gastric cancer patients who underwent radical resection. However, considering the retrospective nature and single-center data of this study, further investigations using prospective and multicenter settings are required to validate our findings.

## Figures and Tables

**Figure 1:** Comparison of disease-free survival (DFS) and overall survival (OS) between the two groups during the 3-year follow-up.

**Table 1:** Clinical data of the study cohorts.

Group	Gender (male/female)	Age		TMN clinical stage			ECOG score		
		<60	≥60	IIIA	IIIB	IIIC	0	1	2
CT (*n* = 45)	33/12	22	23	11	15	19	13	18	14
RCT (*n* = 27)	25/2	11	16	8	10	0	9	12	6
*χ* ^2^		0.451		4.017			0.157		
*p*		0.502		0.134			0.692		

CT: chemotherapy; RCT: radiochemotherapy; ECOG score: Eastern Cooperative Oncology Group score.

**Table 2:** Comparison of acute adverse reactions between the two groups.

Item		Myelosuppression	Gastrointestinal reactions	Neurotoxicity	Liver dysfunction
CT (*n* = 45)	1	20	16	17	13
	2	8	11	10	16
	3	5	0	0	0
	4	0	0	0	0
	5	0	0	0	0
	1~5	31 (73.3%)	27 (60%)	27 (37.78%)	29 (42.22%)
RCT (*n* = 27)	1	17	18	12	7
	2	4	7	5	6
	3	2	0	0	0
	4	0	0	0	0
	5	0	0	0	0
	1-5	23 (85.1%)	25 (92.6%)	17 (62.9%)	13 (48.1%)
*χ* ^2^		0.334	1.387	0.015	0.499
*p*		0.563	0.239	0.903	0.480

CT: chemotherapy; RCT: radiochemotherapy.

## Data Availability

The data used to support the findings of this study are available from the corresponding author upon request.
